# Study on the influencing factors of rural residents’ willingness to classify domestic waste in the context of acquaintance society: An example from Jiangsu Province in Chin

**DOI:** 10.1371/journal.pone.0303167

**Published:** 2024-05-09

**Authors:** Xiaoxu Ma, Nannan Ge

**Affiliations:** 1 Business School, Yangzhou University, Yangzhou, 225127, China; 2 Agricultural Economy in Development Research Institute, Jiangsu Provincial Academy of Agricultural Sciences, Nanjing, 210014, China; King Khalid University, SAUDI ARABIA

## Abstract

Waste classification helps to maximize the recovery of resources, reduce environmental pollution and promote sustainable economic development. To improve the willingness of rural residents to classify waste, based on the background of a rural acquaintance society, this thesis constructed a theoretical model of waste classification cognition, willingness to classify, economic incentives, face consciousness and vernacular identity affecting the willingness of rural residents to classify waste, and put forward seven research hypotheses. With the help of 530 valid surveys of rural residents in Jiangsu Province, the seven hypotheses were verified using structural equation modeling, and the mediating effect of rural residents’ willingness to classify waste was examined using the bootstrap method. The results showed that waste classification awareness, knowledge of waste classification, economic incentives, face-saving concepts and local identity all affected rural residents’ willingness to classify waste, and all were significant at a 0.01 level. They also showed that face-saving concepts and local identity played partial mediating roles. Strategies to improve rural residents’ willingness to classify waste have been proposed, such as multiple incentives to enhance subjective awareness, play the role of face culture in rural areas, strengthen the construction of public culture in rural areas, and improve rural residents’ local identity.

## 1. Introduction

With the rapid development of rural society and economy, the living standards of rural residents are improving, the waste generated in rural areas is becoming increasingly complicated and diversified, and rural areas are facing serious challenges of environmental pollution. At present, the low level of rural domestic garbage classification and the sloppy way in which it is handled have become one of the main source of rural environmental pollution. The destruction of the rural ecological environment and the ever-increasing rural land and water pollution have threatened the physical health of rural residents and brought about a serious impact on their actual lives. The management of rural household waste has become an important issue in improving the rural habitat and comprehensively promoting rural revitalization. China issued the Five-Year Action Program for Improving and Upgrading Rural Habitat (2021-2025) in 2021, which proposes to "accelerate the promotion of classification and reduction of rural domestic waste at source, and to build a system for collecting, transporting, disposing, and recycling rural domestic waste", which marks a new stage of comprehensively upgrading the waste classification and treatment of rural residents. As the first important link, rural residents’ willingness to classify waste directly affects waste classification. Studying the factors influencing rural residents’ willingness to classify waste and proposing countermeasures to improve rural residents’ willingness to classify domestic waste are of great significance for promoting rural waste classification and treatment, maximizing the recovery of resources, reducing environmental pollution and promoting sustainable economic development.

Economist Olson proposed a new perspective on the theory of the logic of collective action, which said "individual rationality leads to collective irrationality."For the sorting of rural household waste, the larger the size of rural collectives, the more likely they are to engage in "fish in troubled waters" and "free-riding" behavior [1]. At home and abroad, research on the factors influencing willingness to separate waste mainly includes two aspects: objective and subjective factors. Studies outside China have mainly focused on the influence of subjective factors on residents’ willingness to classify waste. For example, Babaei et al. studied waste classification behaviors based on survey data in the Abadan area, and found that age, education level, gender and occupation affected their willingness to classify waste [2]. China’s research on the willingness to classify waste mainly focuses on the effects of residents’ environmental perception, literacy, identity, and hardware and software facilities on residents’ willingness to classify waste. Tang’s empirical analysis found that factors such as environmental perception, total household population, literacy, per capita annual income of the household, new occupational farmers, village cadres and party members’ identity affect rural residents’ waste classification willingness and participation level [3]. He pointed out that "in the current Chinese countryside, the ritual order of the acquaintance society and the rule of the elders have long been disintegrated" and turned into a "semi acquaintance society" [4]. Based on the characteristics of the local rural acquaintance society, Liuchi Village utilizes all kinds of social relations to mobilize farmers to participate in waste classification. Jiang found that social relations in an acquaintance society can be used to mobilize rural residents to participate in domestic waste [5].Face consciousness and local identity are significant social characteristics of acquaintances, and there are few studies on the influence of these two aspects on the willingness to separate waste. For example, Shi et al. [6] and Yu et al. [7] analyzed the relationship between face consciousness and the preference and purchase intention of green products; Li F.N. and Zhang J.B. et al. [8] explored the relationship between village identity and participation in environmental governance among farmers; Liu et al. [9] investigated the effect of village sentiment on farmers’ willingness to classify household waste.

Rural China is an "acquaintance society" or "semi acquaintance society", and the "differential order pattern" characterized by the grassroots makes rural residents have special cultural concepts and ritual order, and rural residents value face more than urban residents and have stronger vernacular identity. However, in the existing literature, scholars have only described and analyzed this issue qualitatively, and no scholars have yet quantitatively verified and deeply analyzed the effects of the concept of face and rural vernacular identity on residents’ willingness to participate in domestic waste classification in "acquaintance society" or "semi acquaintance society". The research objectives of this paper are: to explore the influencing factors of rural residents’ willingness to participate in the classification of domestic waste from the perspectives of the concept of face and vernacular identity, using econometric models, coupling countermeasures to improve rural residents’ participation in the classification of domestic waste, further optimizing the current way of treating domestic waste in the countryside, promoting long-term rural domestic waste management, and contributing to the construction of a beautiful countryside that is "ecologically pleasant to live in."

The innovations of this paper are mainly reflected in the following aspects: theoretically, based on the background of the acquaintance society, this paper explores the influence of new variables such as face factor and vernacular identity on rural residents’ willingness to classify waste, which enriches the theory of public goods and the theory of centralized action logic to a certain extent. Based on the findings of the study, this paper proposes to give full play to the role of rural face culture and to strengthen the construction of rural public culture, enhancement of vernacular identity,and other new initiatives to enhance the willingness of rural residents to classify waste, which provides a policy basis for the classification of domestic waste in Jiangsu Province and a reference for the development of domestic waste classification policies in other regions.

This article is organized as follows. First, a review of previous studies on domestic and international rural waste management is presented. A theoretical examination of the paper’s subject was then completed, a theoretical model was built, and research hypotheses were presented. The data collection, choice of key variables, model choice, and analysis of running results are then discussed. Finally, the main conclusions of the study are summarized, and policy recommendations are proposed.

## 2. Theoretical analysis and research hypotheses

Social culture refers to the ideology of a society and its corresponding cultural system and organizational structure, which influences people’s attitudes toward the knowledge and cognition of things, as well as the importance they attach to group recognition, collective belonging, social status, prestige, or dignity. Therefore, based on the special social culture of "acquaintance society" in rural China, this study selected the factors of waste classification cognition, knowledge of waste classification, economic incentives, sense of face, and local identity based on cognitive-behavioral theory, collective action theory, and local identity theory to study their influence on rural residents’ willingness to classify waste.

From cognitive behavioral theory, it is known that individual cognition is the basis of individual will and behavior, and rural residents’ cognition or awareness affects their will and behavior. When exploring the willingness of environmental behavior, Wu empirically found that the higher the level of villagers’ environmental cognition, the higher their willingness to participate in environmental behavior [10]. Xie et al. empirically found that environmental cognition can significantly increase rural residents’WTP for centralized domestic waste disposal,through a study in Shaanxi, Gansu and Henan [11]. Liu et al. empirically found that pollution perceptions positively affect farmers’ willingness to separate waste in a study of 863 households in Shaanxi [9]. Based on the theory of "cognition-attitude-behavior,"Ye et al. empirically analyzed and found that the public’s cognition of haze management had a significant influence on their willingness to pay [12]. Based on this, we propose the following hypotheses:

H1: Waste classification cognition has a positive effect on willingness to classify household waste.

The knowledge of waste classification in this study covers five aspects, including the significance of waste classification, basic standards, laws and regulations and basic knowledge of waste classification skills. Rural residents’ knowledge reserves of waste classification affect their willingness or behavior to a certain extent. Based on the theory of planned behavior and social exchange, Hu and Yu found that environmental knowledge has a significant positive influence on willingness to engage in green behavior [13]. Based on Lewin’s behavioral model, Wang empirically analyzed and found that environmental skills, mainly waste classification skills and other indicators, significantly affect the behavior of farm households [14]. Fan used a two-column model to empirically analyze whether the disclosure of environmental information knowledge can significantly increase the public’s discussion of waste classification and environmental issues, thus influencing the behavior of public participation in environmental protection [15]. Based on this, we propose the following hypothesis:

H2: Knowledge of waste classification has a positive effect on the willingness to classify domestic waste.

Rural domestic waste classification as rural public affairs governance and rural residents participating in the classification of domestic waste will face the dilemma of collective action, so the need for external intervention, which is the most widely discussed two incentives: positive economic incentives, such as the government and village collective subsidies; and negative incentives, such as penalties or mandatory constraints on non-participation in waste segregation. An empirical analysis by Li et al. found that economic incentives,such as subsidies and materials, will reduce the cost of rural residents’ participation in domestic waste classification, thus helping to stimulate the initiative and motivation of rural residents to participate in domestic waste classification [8]. Tang et al., in studying the effects of administrative constraints and economic incentives on the environmental behavior of farm households, found that environmental policies, including environmental administrative policies and environmental economic policies, can motivate farm households to participate in rural environmental governance [16]. Based on this, we propose the following hypothesis:

H3: Economic incentives have a positive effect on the willingness to classify household waste.

Chinese vernacular society is "a network composed of a root of private connections ", which is different from the West, which emphasizes power, and China emphasizes friendship and relationship, and is a society of acquaintances. In this society of acquaintances, face consciousness not only reflects the reciprocal relationship between people but also represents a certain social status, dignity and prestige, which is deeply rooted in the hearts of the Chinese people and is one of the most influential cultural background factors in Chinese behavior. For example, Shi et al. concluded that the stronger a consumer’s ethical face, the more they prefer green products and have more positive prosocial consumption motives [6]. The proposal of China’s ecological revitalization, the construction of an ecologically livable and beautiful countryside, is deeply rooted in people’s hearts, green life, green development, green travel has become a consensus, and rural residents’ recognition of the concept of ecological development is increasing. Based on this, we propose the following hypothesis:

H4: Face consciousness has a positive effect on willingness to classify household waste.

Local identity is the core concept of place theory, which was proposed by Proshansky in 1978 [17], in 1983 introduced local identity into the field of environmental psychology, this paper draws on Proshansky’s explanation and defines local identity as "a part of self-identity, a personal identification with the physical environment, including identification with culture, values, and meanings ", which tends to motivate them to participate in local affairs. China’s vernacular society has its own unique cultural characteristics, rural residents make a living from agriculture, "generations of settlement is the norm ", they have a deeper emotional attachment to their place of residence, the stronger their local identity. Jiang found that all kinds of favor and face-saving relationships through the acquaintance society can promote farmers to develop the habit of consciously classifying household waste [18]. Li et al.found that the higher the village identity of farmers, the more likely they are to participate in environmental governance in the countryside [8]. Liu et al. found that village sentiment has a significant positive effect on farmers’ willingness to categorize household waste [9]. In summary, local identity has a significant influence on rural residents’ participation in environmental governance. Rural residents’ participation in domestic waste classification is an important part of environmental governance, which is an important part of the overall improvement of rural habitats.

H5: Local identity has a positive effect on the willingness to classify household waste.

Place identity includes village emotions and group identity. Village sentiment refers to preference, satisfaction, attachment, and willingness to live permanently in a host village. Group identity refers to identification with the traditional culture and organization of the village. Cognitive behavioral theory points out that cognition can influence individuals’ willingness and behavior, and affective-cognitive theory points out that emotion arises from the cognition and evaluation of environmental stimuli [19]. Local identity, as an emotional-psychological factor of rural residents, can increase the degree of its influence, and local identity can lead to rural residents’ collective consciousness and sense of responsibility for the village, which makes them more willing to carry out the maintenance of the village environment. Liu et al. pointed out that village emotions can strengthen the positive effect of pollution perception on farmers’ willingness to classify waste [9]. Chen and Zhu pointed out that factors such as the herd mentality of rural residents in an acquaintance society can promote their classification of household waste [20]. Based on an empirical study of 12 cities in East China, Wang and Li found that consumers’ emotions toward safe and certified agricultural products played a moderating role in the middle of perception and willingness [19]. Rural residents’ cognition affects their willingness and behavior, while changes in knowledge promote cognitive change [21]. When the knowledge reserve of waste classification is increasing, their awareness of waste classification will gradually improve, and group identity can increase the positive effect of cognition on willingness, so local identity has a mediating effect between knowledge of waste classification and willingness to classify waste.

H6: Local identity has a mediating effect.

H6a: Local identity has a mediating effect between awareness of waste classification and willingness to classify household waste.

H6b: Local identity has a mediating effect between knowledge of household waste classification and the willingness to classify household waste.

H6c: Local identity mediates the relationship between economic incentives and willingness to classify household waste.

At present, China’s rural areas are still in the "acquaintance society" or "semi acquaintance society", and face still represents social status, prestige or dignity in this cultural context. When Wang studied the influence of resource conservation awareness on resource conservation behavior, he pointed out that face consciousness plays a moderating role in the consciousness-situation-behavior model; that is, face consciousness plays a moderating role between cognition and behavior [22]. An increase in individual knowledge can change the cognitive level of an individual, and face consciousness plays a mediating role between cognition and behavior; therefore, face consciousness has a mediating role in the knowledge of waste classification and willingness to participate. Face is a kind of personal social value and achievement, and the government and village collective give some economic subsidies or material incentives to rural residents who do a good job in waste classification and disposal. It is a kind of honor for rural residents; The more collective recognition and praise, the more face-loving people, the more they will actively participate in waste classification work and do a better job by demonstration. The stronger rural residents’ identification with the village collective, the more they want to be recognized by the village collective and pay more attention to the gain or loss of face. To gain better recognition from the group, they are more active and positive in public affairs such as rural waste disposal. In contrast, those with a lower sense of group identity do not care about the views of others, and they will not engage in behaviors that cater to the group for the sake of the so-called loss of face. Based on survey data from Hubei Province, Tang et al. empirically found that face consciousness plays an intermediary role between group identity and centralized waste disposal behavior of rural households [23]. Based on this, we propose the following hypothesis:

H7: Face consciousness has a mediating effect.

H7a: Face consciousness mediates the relationship between economic incentives and willingness to sort waste.

H7b: Face consciousness mediates the relationship between local identity and willingness to categorize waste.

Waste classification cognition (Hypothesis H1) is the premise that knowledge of waste classification (Hypothesis H2) is the foundation, economic incentives (Hypothesis H3) are the external stimulus, and face consciousness (Hypothesis H4, Hypothesis H7) and local identity (Hypothesis H5, Hypothesis H6) are the individual psychological level perceptions. The theoretical basis for Hypotheses H1 and H2 is the classical cognitive-behavioral theory and the research literature of existing scholars; the theoretical basis for Hypothesis H3 is the collective action theory and the research literature of existing scholars; the theoretical basis for Hypotheses H4 and H7 is the research literature of existing scholars; and the theoretical basis for Hypotheses H5 and H6 is the local identity theory and the research literature of existing scholars.

## 3. Research method and data description

### 3.1 Research methodology

#### 3.1.1 Model selection

Structural equation modeling (SEM) is an econometric research method integrating measurement and analysis, which can not only estimate the measurement error of indicator variables but also assess the reliability and validity of related measurements. The traditional regression model can only analyze the direct effect between variables, while the structural equation model can reflect both factor analysis and path analysis, and path analysis can study the influence relationship of multiple independent variables and multiple dependent variables simultaneously. Structural equation modeling mainly consists of two models: measurement model and structural model, in which the measurement model studies the relationship between observed variables and latent variables, and the structural model studies the relationship between each latent variable. Since variables such as awareness of waste classification, knowledge of classification, face factor, and local identity cannot be measured directly and need to be expressed by latent variables and measured by observed variables, with reference to Liu et al. [24], this study chose structural equation modeling for quantitative analysis.

(1) Measurement modeling

Measurement modeling analyzes the relationship between latent variables and the designed questions, that is, observed variables, which are the data obtained by measurement tools such as questionnaires, and latent variables, which are the abstract concepts formed among observed variables. This trait or abstract concept can not be measured directly but is reflected by the data measured by the observed variables. In structural equation modeling, a latent variable must be estimated with more than two observed variables,known as the principle of multiple indicators, and the covariance between different observed variables reflects the common influence of the latent variables.

$$X=\wedge_{x}\xi +\delta$$ (1)

$$Y=\wedge_{Y}\eta +\varepsilon$$ (2)

Where ε is uncorrelated with η, ξ and δ and δ is uncorrelated with ξ and ε with η. ∧_X_ and ∧_Y_ are the factor loadings of the indicator variables (X, Y), while δ and ε are the measurement errors of the exogenous variables, and ξ and η are the exogenous latent variables (dependent variables) and endogenous latent variables (fruit variables), respectively.

(2) Structural modeling

The structural model illustrates the causal relationships between potential variables. The potential variable as the cause can also be called the exogenous potential variable, denoted by ξ, and the potential variable as the effect can also be called the endogenous potential variable, denoted by η. The explanatory variance of the exogenous latent variable on the endogenous latent variable can also be affected by other variables.This is called the disturbance latent variable, denoted by the symbol ζ, which is the disturbance factor or residual value in the structural model. It can also be treated as a path analysis between latent variables in which the regression coefficient in the regression analysis we often talk about is the path coefficient. The relationship between the latent variables can beexpressed as the following structural equation:

η=Bη+Γξ+ζ (3)

B is an (m x m) order matrix, which represents the directional linkage coefficient (regression coefficient) between η variables, and Г is an (m x n) order matrix, which represents the regression coefficient of the effect of ξ variables on η variables.

3.1.2 Theoretical model construction. It is known through cognitive behavioral theory that rural residents’ cognition affects their willingness and behavior, and changes in beliefs and knowledge promote changes in rural residents’ cognition, which in turn promotes changes in rural residents’ willingness to classify household waste. Terry et al. concluded that residents’ experience in classifying household waste has an effect on their classification behavior,that is, residents who have experience in classifying household waste have stronger motivation [25]. Fan et al. found that residents’ trust in waste disposal authorities as well as their perceptions, attitudes, and skills of waste separation have direct or indirect effects on waste separation behavior [26]. China’s rural areas are still in an "acquaintance society" or "semi acquaintance society," and rural residents, based on face-saving, seek recognition from the village community and maintain their prestige in the village, are more inclined to choose behaviors that have the common values of the village, and thus are more willing to participate in domestic waste classification. Therefore, when studying the influencing factors of rural residents’ willingness to classify waste, this study mainly explores the influence of controllable factors and their influence paths. The specific theoretical model is shown in Fig 1.

**Fig 1:** Structural equation model of domestic waste classification willingness.

### 3.2 Data collection

The data for this study was obtained from micro-surveys, using the rural areas of six districts and counties under the jurisdiction of Lianyungang City, Jiangsu Province, as the object of research.First, a number of townships were randomly selected from six districts and counties, and then a number of villages were randomly selected in the townships. Five to six researchers were selected from each district and county, whose specialties were related to agricultural economic management or who had previous experience in rural survey.A total of 550 questionnaires were distributed and 530 valid questionnaires were recovered, with a validity rate of 96.4%. Among them, 85 questionnaires were collected from Haizhou District (validity rate 97.7%), 93 from Lianyun District (validity rate 96.9%), 106 from Ganyu District (validity rate 96.4%), 81 from Donghai County (validity rate 96.4%), 79 from Gandong County (validity rate 95.2%), and 86 from Ganyun County (validity rate 95.6%).

### 3.3 Selection of core variables

The theory of rational behavior holds that the will to act is formed by an individual’s subjective attitude and subjective norms, and these factors determine whether a person finally performs a certain behavior. In other words, residents’ behavioral attitudes and subjective tendencies determine whether they engage in certain behaviors. Based on this, this study mainly explores the factors influencing rural residents’ willingness to classify domestic waste from the perspective of controllable factors based on the background of the acquaintance society, so the following core variables were selected.

This article sets the following variables: "environmental cognition" in the previous literature, and referring to the construction of "environmental cognition" indicators by Wang [14,21], this article sets the following variables: "waste sorting is beneficial to environmental protection in the village," "waste sorting is beneficial to residents’ health," "waste sorting can hinder the spread of diseases," and "waste sorting can prevent the pollution of arable land and soil," the four indicators to measure the "cognition of waste classification," According to the three indicators of "environmental knowledge" classified by Wang [14] and the construction of indicators of "environmental knowledge" by Meng [27]. In this study, we set "I clearly know the significance of waste classification", "I clearly know the specific standards of waste classification", "I know the laws, regulations,or policies related to waste classification", "I can skillfully classify waste" and "I am able to classify waste after mastering the waste classification standards", and the five indicators to measure waste classification knowledge. According to the three indicators of "economic incentives" classified by Wang [14] and the construction of "economic incentives" by Xiang [28]. In this study, we set up four indicators to measure "economic incentives", namely, "sorting waste to make it easier to sell for profit", "incentives from the village collectives help us to sort waste", "subsidies from the government help us to sort waste", and "appropriate penalties for failing to sort waste help us to sort waste". The values of "waste classification cognition,” "waste classification knowledge" and "economic incentives" are shown in Table 1.

**Table 1:** Measurement index setting and assignment description.

variable	Indicator name	Variable assignment	Mean	S.D
GC: Cognition of waste sorting	GC1 Separation of waste is beneficial to the environmental protection of the village.	Strongly Disagree = 1,Not Really Agree = 2, Fairly Agree = 3, Quite Agree = 4, Strongly Agree = 5	4.43	0.897
	GC2 Separating waste is good for the health of residents.	Strongly Disagree = 1,Not Really Agree = 2, Fairly Agree = 3, Quite Agree = 4, Strongly Agree = 5	4.45	0.882
	GC3 Sorting waste can hinder the spread of disease.	Strongly Disagree = 1,Not Really Agree = 2, Fairly Agree = 3, Quite Agree = 4, Strongly Agree = 5	4.40	0.954
	GC4 Sorting waste prevents contamination of arable soil.	Strongly Disagree = 1,Not Really Agree = 2, Fairly Agree = 3, Quite Agree = 4, Strongly Agree = 5	4.38	0.958
GK: Knowledge of waste sorting	GK1 I know exactly what it means to separate waste.	Strongly Disagree = 1,Not Really Agree = 2, Fairly Agree = 3, Quite Agree = 4, Strongly Agree = 5	4.09	1.082
	GK2 I am well aware of the specific criteria for waste separation.	Strongly Disagree = 1,Not Really Agree = 2, Fairly Agree = 3, Quite Agree = 4, Strongly Agree = 5	3.68	1.255
	GK3 I know the laws and regulations or policies related to waste separation.	Strongly Disagree = 1,Not Really Agree = 2, Fairly Agree = 3, Quite Agree = 4, Strongly Agree = 5	3.60	1.288
	GS1 I can skillfully sort waste.	Strongly Disagree = 1,Not Really Agree = 2, Fairly Agree = 3, Quite Agree = 4, Strongly Agree = 5	3.59	1.253
	GS2I was able to separate my waste after I mastered the criteria for separating waste.	Strongly Disagree = 1,Not Really Agree = 2, Fairly Agree = 3, Quite Agree = 4, Strongly Agree = 5	4.09	1.036
EI:Economic incentives	EI1 waste is categorized in order to make it easier to sell the waste for profit.	Strongly Disagree = 1,Not Really Agree = 2, Fairly Agree = 3, Quite Agree = 4, Strongly Agree = 5	3.49	1.333
	EI2 The incentives from the village collectives help us to categorize our waste.	Strongly Disagree = 1,Not Really Agree = 2, Fairly Agree = 3, Quite Agree = 4, Strongly Agree = 5	4.02	1.057
	EI3 Government subsidies help us to segregate waste.	Strongly Disagree = 1,Not Really Agree = 2, Fairly Agree = 3, Quite Agree = 4, Strongly Agree = 5	4.11	1.018
	EI4 Giving appropriate penalties for not separating waste properly helps us to separate waste.	Strongly Disagree = 1,Not Really Agree = 2, Fairly Agree = 3, Quite Agree = 4, Strongly Agree = 5	3.96	1.096

The results of the factor analysis showed that the KMO value of awareness of waste sorting was 0.822, the KMO value of knowledge of waste classification was 0.860, the KMO value of economic incentives was 0.802,the KMO value of the three latent variables met the requirements,the Cronbach’s α value of awareness of waste sorting was 0.947, the Cronbach’s α value of knowledge of waste classification was 0.935, the Cronbach’s α value of economic incentives was 0.846, and the reliability of the Cronbach’s α values met the requirements.

Face consciousness is a unique Chinese cultural psychology, social status, self-esteem and prestige that involves many fields such as sociology, psychology, and political science. By drawing on Zhang dimensions of "wanting to lose face" and "fearing to lose face" [29], and the method of face measurement proposed by Tang et al., this paper sets up five related questions, specifically "waste classification can make me praised," "If others do a good job of waste classification, but I don’t do a good job to make me lose face," "My position in the village is very important," "I care a lot about honorary titles such as ’Model Farmer for waste Separation"and "I care a lot about what others think and say about me." Many scholars at home and abroad divide "local identity" into different dimensions for measurement according to their needs, and the author draws on Yuan and Chen’s division of dimensions [30], set "I agree with the traditional customs of this village", "I think such a form of organization in the countryside is very important", "I feel satisfied living in the village", "I would like to live in this village forever", "I would feel sad if I were to move away from this village"and "personal relationships in the village are important to me",and the six indicators to measure "local identity". The values of "face consciousness" and "local identity" are listed in Table 2.The results of the factor analysis showed that the KMO value for face consciousness was 0.870, and the KMO value for local identity was 0.893.The Cronbach’s alpha value of face consciousness was 0.906, and that of place identity was 0.924, which was in line with the requirements.

**Table 2:** Face Consciousness and local identity measurement index setting and assignment description.

Variables	Indicator name	Variable assignment	Mean	S.D
FC:face consciousness	FC1 Separating waste can get me praised.	Strongly Disagree = 1,Not Really Agree = 2, Fairly Agree = 3, Quite Agree = 4, Strongly Agree = 5	3.60	1.153
	FC2 I have an important position in the village.	Strongly Disagree = 1,Not Really Agree = 2, Fairly Agree = 3, Quite Agree = 4, Strongly Agree = 5	3.19	1.231
	FC3 If someone else is doing a good job of separating waste, it makes me lose face if I don’t do a good job.	Strongly Disagree = 1,Not Really Agree = 2, Fairly Agree = 3, Quite Agree = 4, Strongly Agree = 5	3.70	1.090
	FC4 I care a lot about what people think and say about me.	Strongly Disagree = 1,Not Really Agree = 2, Fairly Agree = 3, Quite Agree = 4, Strongly Agree = 5	3.66	1.092
	FC5 I am very concerned about the honorary title of "Model Farmer in waste Sorting".	Strongly Disagree = 1,Not Really Agree = 2, Fairly Agree = 3, Quite Agree = 4, Strongly Agree = 5	3.59	1.139
LI:local identity	LI1 I agree with the traditional customs of our village.	Strongly Disagree = 1,Not Really Agree = 2, Fairly Agree = 3, Quite Agree = 4, Strongly Agree = 5	3.80	1.020
	LI2 I think it’s important for rural areas to be organized in this way.	Strongly Disagree = 1,Not Really Agree = 2, Fairly Agree = 3, Quite Agree = 4, Strongly Agree = 5	3.99	.957
	LI3 I feel content living in the village.	Strongly Disagree = 1,Not Really Agree = 2, Fairly Agree = 3, Quite Agree = 4, Strongly Agree = 5	3.86	1.009
	LI4 I would like to live in this village all the time.	Strongly Disagree = 1,Not Really Agree = 2, Fairly Agree = 3, Quite Agree = 4, Strongly Agree = 5	3.75	1.109
	LI5 If I were to move away from this village, I would feel very sad.	Strongly Disagree = 1,Not Really Agree = 2, Fairly Agree = 3, Quite Agree = 4, Strongly Agree = 5	3.83	1.073
	LI6 Personal relationships in the village are important to me.	Strongly Disagree = 1,Not Really Agree = 2, Fairly Agree = 3, Quite Agree = 4, Strongly Agree = 5	3.87	1.044

## 4. Data analysis and main findings

### 4.1 Verification of structural equation modeling

#### 4.1.1 Modification of structural equation modeling

There are many indicators of model fit: through the first empirical evidence, the indicators will appear more out of the standard range, resulting in the model not meeting the standard, to obtain a better fit that needs to be constantly adjusted to the model. The approach taken in this study is to continuously adjust and improve the fit of the model through the model covariance;there is a significant positive covariance relationship (correlation) between knowledge of waste sorting and perception of waste sorting, with a standardized path coefficient value of 0.607>0, significant at the 0.01 level (z=11.969, p=0.000), and there is a significant positive covariance relationship (correlation) between financial incentives and perception of waste sorting, with a standardized path coefficient value of 0. 461> 0, significant at the 0.01 level (z=9.658, p=0.000); and there is a significant positive covariance (correlation) between economic incentives and knowledge of waste classification, with a standardized path coefficient value of 0. 510>0, significant at the 0.01 level (z=10.476, p=0.000). Therefore, covariance relationships between knowledge of waste classification and perception of waste classification, financial incentives and perception of waste classification, and financial incentives and knowledge of waste classification were established.

#### 4.1.2 Fit of the structural equation model

Structural equation modeling is mainly used to test whether the proposed research hypothesis can be supported by empirical data.Before analyzing the results of structural equation modeling, the fitness of the model needs to be analyzed. The fit of the model was tested using AMOS 23.0, mainly using the following three types of indicators. The first is the absolute fit index. For example, the chi-square value (χ^2^) indicates how well the overall causal path diagram of this model matches the actual data, but because the chi-square value is very sensitive to the size of the sample;that is, the larger the number of samples, the more the chi-square tends to reach significance, which makes the theoretical model the more probable it is to be rejected, scholars usually use the ratio of the chi-square value to the value of the free value as an indicator of the model’s fit, that is, CMIN/DF. The second indicator is the incremental fit indicator. This type of index is also constrained by the sample capacity, has higher stability when using the great likelihood estimation, and can cope with more complex models, but the estimation results have larger variation values, that is, larger standard deviation, including the NFI, RFI, IFI, CFI, and TLI. The third was the streamlined fit index. Third, we used a streamlined fit index. Unlike absolute and incremental fit indicators, such indicators are less strongly constrained by the sample capacity, are suitable for simple estimation models, and can also be used for comparison between different models, including PNFI and PCFI. The test results of each fitness were derived through adjustment, and the details are shown in Table 3; GFI, CFI, TLI, NFI and IFI were all greater than 0.9, χ^2^/DF = 2.08, and RMSEA < 0.05.

**Table 3:** Model fitting index.

Common indicators	Standard criteria	Value	Common indicators	Standard criteria	Value
df	-	2	NNFI	>0.9	0.925
p	>0.05	0.000	TLI	>0.9	0.925
χ^2^/df	<3	2.08	AGFI	>0.9	0.896
GFI	>0.9	0.988	IFI	>0.9	0.990
RMSEA	<0.10	0.083	RMR	<0.05	0.019
CFI	>0.9	0.990	SRMR	<0.1	0.019
NFI	>0.9	0.989	RMSEA 90% CI	-	0.078~ 0.181

There are many model-fitting indicators, and it is usually only necessary to focus on the chi-square degrees of freedom ratio, GFI, RMSEA, RMR, CFI, NFI, NNFI, and NNFI in total seven indicators. Therefore, the results in the table show that the theoretical model fits the sample data well.

### 4.2 Path analysis of structural equation modeling

In this study, according to the theoretical model constructed previously, Amos 23.0 was used to test the influence of each latent variable on the willingness to classify household waste, and at the same time, the interrelationships between the latent variables were verified.

Waste classification cognition, knowledge of waste classification, economic incentives, face consciousness and local identity have a significant effect on rural residents’ willingness to classify waste. Knowledge of waste classification positively affects rural residents’ willingness to classify waste, with a standardized path coefficient value of 0.064>0, which is significant at the level of 0.01. Knowledge of waste classification positively affects rural residents’ willingness to classify waste, with a standardized path coefficient value of 0.291>0, which is significant at the level of 0.01. Economic incentives positively affect rural residents’ willingness to classify waste, with a standardized path coefficient value of 0.169>0, which is significant at the level of 0.01.Face consciousness positively affects rural residents’ willingness to classify waste, with a standardized path coefficient value of 0.102>0, which is significant at the level of 0.01.Local identity positively affects rural residents’ willingness to classify waste, with a standardized path coefficient value of 0.293>0, which is significant at the level of 0.01.

The standardized path coefficient value for the effect of economic incentives on the concept of face is 0.313>0, and this path shows a significance level of 0.01, indicating that economic incentives have a significant positive effect on the concept of face and the effect of local identity on the concept of face. The standardized path coefficient value for the value of 0.472>0, and this path shows a significance level of 0.01, thus indicating that the relationship between local identity has a significant positive influence on face perception.(The data are presented in Table 4)

**Table 4:** Summary of model regression coefficients.

Path X→Y	Unstandardized path coefficients	SE	z (CR Value)	p	Standardized path coefficients
EI→FC	0.313	0.038	8.254	**	0.301
LI→FC	0.472	0.038	12.433	**	0.412
GC→LI	0.050	0.041	1.196	0.232	0.041
GK→LI	0.381	0.043	8.893	**	0.281
EI→LI	0.358	0.038	9.353	**	0.318
GC→GW	0.084	0.033	2.511	**	0.064
GK→GW	0.310	0.037	8.417	**	0.291
EI→GW	0.189	0.035	5.386	**	0.169
FC→GW	0.101	0.036	2.807	**	0.102
LI→GW	0.303	0.039	7.792	**	0.293
GC→GC1	1.000			**	1.000
GC→GC2	1.009	0.023	44.407	**	1.009
GC→GC3	0.980	0.032	30.616	**	0.980
GC→GC4	1.001	0.031	32.148	**	1.001
GK→GK1	1.000			**	1.000
GK→GK2	1.502	0.066	22.774	**	1.502
GK→GK3	1.528	0.068	22.338	**	1.528
GK→GK4	1.501	0.066	22.584	**	1.501
GK→GK5	1.105	0.058	19.054	**	1.105
EI→EI1	1.000			**	1.000
EI→EI2	1.193	0.057	20.888	**	1.193
EI→EI3	1.267	0.060	21.007	**	1.267
EI→EI4	0.904	0.075	12.078	**	0.904
FC→FC1	1.000			**	1.000
FC→FC2	0.966	0.038	25.653	**	0.966
FC→FC3	0.954	0.038	25.089	**	0.954
FC→FC4	0.914	0.047	19.308	**	0.914
FC→FC5	0.900	0.043	21.002	**	0.900
LI→LI1	1.000			**	1.000
LI→LI2	1.041	0.043	24.370	**	1.041
LI→LI3	1.072	0.045	23.905	**	1.072
LI→LI4	1.030	0.039	26.092	**	1.030
LI→LI5	0.859	0.040	21.503	**	0.859
LI→LI6	0.837	0.044	18.826	**	0.837
GW→GW1	1.000			**	1.000
GW→GW2	0.865	0.029	29.532	**	0.865
GW→GW3	1.079	0.036	30.277	**	1.079
GW→GW4	1.011	0.047	21.457	**	1.011

Note.

→ indicates a path relationship

** indicates that P has a value less than 0.01.

The impact of waste classification cognition on local identity, this path does not show significance, thus indicating that waste classification cognition does not have an impact on local identity; waste classification knowledge on local identity, the standardized path coefficient value of 0.381>0, and this path shows 0.01 level of significance, thus indicating that knowledge of waste classification has a significant positive impact on local identity; Economic incentives on local identity, the standardized path coefficient value is 0.358>0, and this path shows 0.01 level of significance, thus indicating that economic incentives have a significant positive impact on local identity.(The data are presented in Table 4)

### 4.3 Analysis of the results of the mediating role

Based on the research hypothesis above, face consciousness and local identity play a mediating role in the influence of rural residents’ willingness to participate in waste sorting. This study considers personal characteristics such as gender, age, education and physical health as control variables and uses the bootstrap sampling method to test the mediating role. The basic theoretical mathematical model for the test of the mediating role is shown in Fig 2.

**Fig 2:** Mathematical model diagram of the basic theory for testing the mediation effect where c is the total effect of X on Y, c’is the direct effect, and a*b is the mediating effect.

#### 4.3.1 Analysis of the mediating effect of local identity

The mediation effects model was divided into three regression models. Model 1 constructs a regression model of independent variable X and dependent variable Y, that is, the regression of waste classification cognition and willingness to participate in waste classification; Model 2 refers to the regression model of independent variable X and mediator variable M, that is, the regression of waste classification cognition and local identity; Model 3 refers to the regression model of independent variable X and mediator variable M together with dependent variable Y,that is, the regression of waste classification cognition and local identity together with dependent variable Y. knowledge and local identity together with the willingness to participate in waste classification regression. Model 4 refers to the regression of knowledge of waste classification and willingness to participate in waste classification; Model 5 refers to the regression of knowledge of waste classification and local identity; Model 6 refers to the regression of knowledge of waste classification and local identity together with willingness to participate in waste classification; Model 7 refers to the regression of economic incentives and willingness to participate in waste classification; Model 8 refers to the regression of economic incentives and local identity; Model 9 refers to the regression of economic incentives and local identity together with the regression of willingness to participate in waste classification. The results of the specific analysis are listed in Table 5.

**Table 5:** Analysis results of the mediating role of local identity.

Varibles	Model 1	Mode 2	Mode 3	Mode 4	Mode 5	Mode 6	Mode 7	Mode 8	Mode 9
	B (Unstandardized regression coefficients)								
Constant	-1.202*	-1.114**	-0.554*	-0.621*	-0.584	-0.349	-1.090**	-0.964**	-0.589*
Gender	0.135	0.121	0.064	0.096	0.085	0.057	0.119	0.096	0.069
Age	0.001	0.008*	-0.004	0.001	0.008*	-0.003	0.001	0.008*	-0.003
Cultural level	0.069	-0.044	0.095**	0.049	-0.063	0.079*	0.066	-0.052	0.093**
Health	0.186**	0.187**	0.077*	0.07	0.083	0.032	0.164**	0.162****	0.080*
GC	0.501**	0.441**	0.245**						
GK				0.668*	0.599**	0.389****			
EI							0.593**	0.572**	0.296**
LI			0.582**			0.465**			0.520**
R ^2^	0.313	0.231	0.573	0.483	0.375	0.618	0.41	0.36	0.583
Adjusted R ^2^	0.306	0.224	0.568	0.478	0.369	0.614	0.405	0.353	0.579

Note.

*Represents significance at the level 0.05

**represents significance at the level of 0.01.

Through empirical analysis, we analyze whether the total effect, direct effect and indirect effect of local identity on waste classification cognition (GC) and willingness to participate (GW), waste classification knowledge (GK), willingness to participate (GW), economic incentives (EI) and willingness to participate (GW) exist, and then verify whether local identity plays a mediating role, and summarize the paths of each factor. The results of the validation of the mediating role of local identity are shown in Table 6. A and b are significant in the table, and c’ is significant, and a*b and c’ have the same sign . Then,it is a partial mediating role, so that local identity plays a partially mediating role between the awareness of waste sorting and the willingness to participate in waste sorting. Rural residents’ knowledge and evaluation of waste classification can stimulate their emotions towards the village and their identification with the group, thus making them more willing to participate in waste classification. Rural residents’ knowledge of waste classification and economic incentives can increase their sense of local identity, thereby increasing their willingness to participate.

**Table 6:** The results of the mediating role test of local identity.

Term	c	a	b	a*b	a*b	a*b	C’
	Total effect			Intermediation effect	Boot SE	95% Boot CI	Direct effect
GC=>LI=>GW	0.501**	0.441**	0.582*	0.257	0.001	0.199~0.311	0.245**
GK=>LI=>GW	0.668**	0.599**	0.465**	0.278	0.001	0.222~0.339	0.389**
EI=>LI=>GW	0.593**	0.572**	0.520**	0.298	0.001	0.242~0.355	0.296**

Note.

* Represents significance at the level 0.05

** represents significance at the level of 0.01.

#### 4.3.2 Mediating effect analysis of face consciousness

The mediating effect model is divided into three types of regression models:Model 1 constructs the regression model of independent variable X and dependent variable Y,that is, the regression of economic incentives and the willingness to participate in waste sorting; Model 2 refers to the regression model construction of the independent variable X and the mediating variable M, that is, the regression of economic incentives and face consciousness; Model 3 refers to the regression model construction of the independent variable X and the mediating variable M together with the dependent variable Y, that is, the regression of economic incentives and face consciousness together with the regression of the willingness to participate in waste classification; Model 4 is the regression of local identity and the willingness to participate in waste classification; Model 5 is the regression of local identity and face consciousness; Model 6 is the regression of local identity and face consciousness together with the willingness to participate in waste classification. The results of the specific analysis are presented in Table 7.

**Table 7:** Analysis results of the mediating role of face consciousness.

Varibles	Model 1	Mode 2	Mode 3	Mode 4	Mode 5	Mode 6
	B (Unstandardized regression coefficients)					
Constant	-1.090**	-1.108**	-0.699*	-0.626*	-0.713*	-0.461
Gender	0.119	-0.137	0.167*	0.094	-0.153*	0.130*
Age	0.001	0.008*	-0.002	-0.005	0.002	-0.006
Cultural level	0.066	-0.003	0.067	0.120**	0.049	0.108**
Health	0.164**	0.254**	0.074	0.074	0.175**	0.034
GC	0.593**	0.577**	0.390**			
GK				0.691**	0.636**	0.544**
EI			0.353**			0.231**
LI	0.41	0.393	0.486	0.527	0.457	0.556
R ^2^	0.405	0.387	0.48	0.522	0.452	0.55

Note.

* Represents significance at the level 0.05

** represents significance at the level of 0.01.

Through empirical analysis, we analyze whether the total, direct and indirect effects of face consciousness exist in terms of economic incentives (EI) and willingness to participate (GW), local identity (LI) and willingness to participate (GW). We then verify whether face consciousness plays a mediating role and summarize the path of each factor. The results of the validation of the mediating role of face consciousness are presented in Table 8. In the table, a and b are significant and c’ is significant, and a*b and c’ have the same sign, indicating a partial mediating role; therefore, face consciousness plays a partial mediating role between economic incentives and the willingness to participate in waste sorting. When carrying out waste classification work, the village group’s incentives, government subsidies and appropriate punishments help to improve the face consciousness of rural residents, thus increasing their willingness to participate in waste classification. The higher the rural residents’ emotional and group identification with the village, the more they pay attention to the gain or loss of face. In order to maintain their face, they behave more proactively to cater to the needs of the group in public affairs such as rural waste disposal.

**Table 8:** The results of the mediation test of face consciousness.

Term	c	a	b	a*b	a*b	a*b	C’
	Total effect			Intermediation effect	Boot SE	95% Boot CI	Direct effect
EI=>FC=>GW	0.593**	0.577**	0.353**	0.204	0.001	0.145~0.270	0.390**
LI=>FC=>GW	0.691**	0.636**	0.231**	0.147	0.001	0.085~0.214	0.544**

Note.

* Represents significance at the level 0.05

** represents significance at the level of 0.01.

## 5. Conclusions and recommendations

### 5.1 Conclusions

Based on the theories of public goods and rational behavior, this study uses structural equation modeling to study how face consciousness, local identity, and economic incentives affect rural residents’ willingness to classify waste using research data related to waste classification in Jiangsu Province,China. The Bootstrap method was used to test whether there was a mediating effect on rural residents’ willingness to classify waste and to explore the path of the mediating effect. The conclusions of this study are as follows:

1. Cognition of waste classification, knowledge of waste classification,economic incentives, face consciousness and local identity had a significant positive effect on rural residents’ willingness to classify waste. Government subsidies, village collective incentives and penalties increase rural residents’ willingness to separate household waste. The higher the awareness of waste classification, the higher the knowledge of waste classification, the stronger face consciousness,the higher the sense of local identity of rural residents, and the more willing they are to participate in the treatment of domestic waste classification.
2. Face consciousness and local identity played a partially mediating role. Face consciousness partially mediates the relationship between economic incentives and willingness to classify household waste, local identity and willingness to classify household waste. Local identity plays a partially mediating role between the perception of waste classification and the willingness to classify household waste, knowledge of waste classification and the willingness to classify household waste, and economic incentives and the willingness to classify household waste.

### 5.2 Policy recommendations

First, it improves the system of classification and governance and provides various incentives to promote the awareness of the main body. domestic waste in rural areas belongs to public goods to avoid the emergence of "free-riding" behavior. The government should issue relevant policies on rural waste classification and management in a timely manner, and establish and improve relevant laws and regulations. Village collectives should formulate village incentives, such as direct subsidies, material incentives, such as rewards in kind, or honorary incentives,such as awarding honorary titles and giving village concessions, to enhance their sense of honor and pride in participating in rural public services. Establish a village punishment system, through criticism and education, on the village black list, cancel village preferences and other measures, restrain rural residents of waste classification behavior, and actively participate in the work of waste classification in the capacity of the village master.

Second, it plays the role of village face culture in promoting effective waste classification governance. Actively give full play to the culture of face in rural China, and improve the level of environmental awareness of rural residents according to local conditions and village conditions, so as to promote the willingness of rural residents to participate in waste classification with their sense of "love of face". Through a variety of publicity channels, the good deeds of active participation in waste classification will penetrate the hearts of rural residents. Regularly carrying out skills training in waste classification improves the practical skills of rural residents in waste classification, gives high recognition and praise to those who perform well in the training process, and carries out spiritual rewards and material rewards to improve the willingness of residents to participate in and enhance the ability to classify household waste, so as to enhance the substantive effect of the management of household waste classification.

Third,we should strengthen the construction of a rural public culture and improve the local identity of rural residents. Improve the infrastructure for cultural construction, provide a space for mutual exchange and learning of rural cultural knowledge, and improve the relevant knowledge and cultural levels of rural residents. Inheriting an excellent local culture, strengthening the sense of village identity, and improving the sense of participation of the main body. According to the traditional customs of the village plus innovative factors, the village collectives take the lead in organizing a variety of enjoyable cultural activities to stimulate their interest in participating in village public affairs, enhance the sense of identity of rural residents in the village, and through the recognition of the village organization, increase their willingness to participate in waste classification, promote the waste classification work in the area, and give play to their role in improving the human habitat and building a beautiful and ecologically livable countryside.

## Discussion

First, the management of domestic waste classification is systematic, and there are many factors affecting the willingness of rural residents to classify. Because of the subjectivity of the selected research angle factors, the next step can be explored on the basis of objective factors, such as the infrastructure in rural areas, the government and the village collectives of publicity. Whether waste classification can be successfully carried out in a region, in addition to focusing on the willingness of rural residents to classify waste, we should also focus on the influence of external objective factors.

Second,rural residents in China tend to live together in concentrated groups, and a society with acquaintances is a common state of affairs. The face factor and local identity are aspects that villagers particularly value and have a strong influence on rural household waste sorting.This cultural context does not vary much between different regions of China, making it representative of the situation in China.China’s culture is very different from that of the rest of the world, since this study was conducted based on China’s acquaintance society. The findings have general applicability in China, but not so much in other cultures. If possible, the factors influencing rural residents’ willingness to categorize waste in other cultures should be further explored in the future.

## Supporting information

S1 Data (XLS)
